RETRACTED

# Environmental dust removal from inclined hydrophobic glass surface: avalanche influence on dynamics of dust particles

**DOI:** 10.1039/c8ra07503d

**Published:** 2018-10-02

**Authors:** Bekir Sami Yilbas, Abdullah Al-Sharafi, Haider Ali, Nasser Al-Aqeeli, Hussain Al-Qahtani, Fahad Al-Sulaiman, Numan Abu-Dheir, Ghassan Abdelmagid, Ali Elkhazraji

**Affiliations:** Center of Excellence in Renewable Energy, King Fahd University of Petroleum & Minerals Dhahran Saudi Arabia bsyilbas@kfupm.edu.sa; Mechanical Engineering Department, King Fahd University of Petroleum & Minerals Dhahran Saudi Arabia

## Abstract

The removal of environmental dust particles from optically transparent glass surfaces is considered, and the dynamics of the dust particles on the inclined hydrophobic glass surface is examined. The glass surfaces are coated by functionalized nano-sized silica particles to create a hydrophobic wetting state on the surface. A thin layer of environmental dust particles, collected from the local area of Dammam in the Kingdom of Saudi Arabia (KSA), is deposited on the surface while mimicking the dust accumulation on the surfaces in the dusty days of KSA. In order to increase the removal rate of the dust particles from the inclined hydrophobic glass surfaces, high density particles, which are higher than the density of the dust particles, are locally distributed on the dust particle-deposited surface while generating the avalanche influence on the inclined surface. The motion of the dust and high density particles on the inclined surface is monitored using a high speed camera. The predictions of the dust particles' acceleration and velocity are compared to those obtained from the high speed camera data. It is found that the predictions of velocity and acceleration of the dust particles agree well with the experimental data. Local insertion of the high density particles generates avalanche influence on the inclined surface while initiating the removal of the dust particles from the hydrophobic surface at small inclination angles. The size of the area where the dust particles are removed from the inclined surface increases with enlarging coverage area of the high density particles. The dust-removed surface, under the avalanche influence, improves the UV-visible transmittance of the hydrophobic glass.

## Abstract 2

The removal of environmental dust particles from optically transparent glass surfaces is considered, and the dynamics of the dust particles on the inclined hydrophobic glass surface is examined.

## Introduction

Optical transparency of glasses remains critical in dusty environments. This is particularly important in regions where dust storms are affective due to the recent climate change. Dust accumulation has multi-fold effects on surfaces, and this is particularly true in humid ambient air.^1^ In general, dust particles consist of various elements, and the particle composition changes from region to region depending on the regional geological characteristics.^2^ However, some dust particles can suspend in air and are carried over long distances by strong winds. These airborne particles cover the landscape surfaces when the influence of wind power diminishes. This contributes to dust particle accumulation on surfaces, which is mostly observed after the dust storms. Many methods and techniques have been developed to remove dust particles from surfaces.^3–5^ However, some of these methods and techniques require either clean water,^3^ compressed air^4^ or mechanical brushing,^5^ and excessive energy use becomes unavoidable in these processes. Because of the scarcity of clean water and shortage of electric power, adopting a self-sustainable mechanical method for dust particle removal becomes important, which is particularly true in the areas where electrical power is not readily available. Utilizing the gravitational force through tilting the dusty surfaces can contribute to the dust removal from surfaces. However, the pinning forces, some of which include the force due to dust particle adhesion on the surface, interlocking and interfacial forces among the accumulated dust particles on the surface, and frictional force play an important role in the dynamics of the dust particles on surfaces. Size, shape, density, and electrostatic charge variation among the dust particles become key factors in determining the pinning forces. The proper arrangement of the factors affecting the dynamics of dust particles can create the avalanche effect on the surface while enhancing dust particle removal from the surface. Consequently, investigation of the dust particle dynamics on inclined surfaces towards generating the self-cleaning effect on the surfaces becomes essential.

RETRACTED

In general, sustainable self-cleaning requires a hydrophobic wetting state on surfaces.^6–8^ Hydrophobic wetting state is mainly associated with the surface texture composed of hierarchically distributed micro/nano pillars and low surface free energy. The desired surface texturing can be accomplished by many methods, including chemical processing,^9^ laser ablation,^10^ mechanical grinding/machining,^11^*etc.* However, texturing of optically transparent surfaces requires special care towards keeping the optical properties, such as UV visible transmittance, reflection, and absorption. Surface texturing modifies the optical characteristics of the surface because of scattering and diffusion of the incident UV-visible radiation by the textured pillars and fibrils. This has significant influence on the photovoltaic device performance. Although impregnating the textured surface with a liquid matching the optical properties, such refractive index and extinction coefficient, improves the optical transmittance, the wetting state of the surface changes significantly because of the liquid encapsulation of the textured surface.^12^ Hence, one-step surface texturing with improved optical transmittance has become in demand for photovoltaic applications. On the other hand, recent changes in climate cause dust storms around the globe, and the dust accumulation on optically transparent surfaces greatly influences the performance of energy harvesting devices such as photovoltaics, thus reducing the device performance significantly.^13^ This is mainly because of the reduced transmittance of UV-visible radiation that reaches the active device surface and the excessive surface heating because of the increased absorption of solar radiation by the dust particles. In general, the dust particles comprise various elements, including alkaline and alkaline earth metals. In humid ambient air, water condensates on dust particles, and some alkaline and alkaline earth metal compounds can dissolve in the water condensate.^14^ This forms a chemically active fluid, which dispenses and wets the optically active surface under the gravitational potential energy.^15^ A layer is formed gradually on the surface *via* accumulation of the dispensed liquid; however, as the liquid layer dries, crystal structures are formed from the residues of the liquid film.^14^ These crystals strongly adhere on the surface and form an intermediate bonding layer between the surface and the dust particles. The efforts required to clean such surfaces become extremely difficult and require energy-intensive processes. This situation may also be observed during the cleaning of such surfaces with a water droplet or water film. In order to avoid the formation of an active liquid layer on the surface, the process involving a dry cleaning becomes fruitful. Several methods have been introduced for dry cleaning of such surfaces. Some of these include electrostatic repulsion of the dust particles,^15^ mechanical brushing of the surfaces,^5^*etc.* Most of these processes involve energy-intensive cleaning and may require additional equipment, which could be permanently installed on the sites. One of the methods for self-cleaning of optical surfaces is creating an avalanche effect on the surface while removing a large amount of mass of the dust particles. To initiate such process, two important conditions need to be satisfied. These include: (i) facilitating the mechanism for the particles to move down on the surface under the influence of gravitational potential energy, and (ii) generating density differences in the dust particles so that the heavy particles initiate rolling/sliding on the surface under the influence of gravitational potential energy. Although several research studies have been carried out to examine the flow on surfaces under the avalanche influence,^16–19^ most of these studies are limited with the consideration of either large particles, such as rocks and snowfalls over mountains and hills,^16–18^ and particles in rotating drums.^19^ Inclination of the optical surfaces may not involve energy-intensive processes, and this arrangement can be used for self-cleaning of surfaces from the dust particles; in this case, large amounts of the dust particles can be removed *via* generating the avalanche influence on the inclined surface.

RETRACTED

On the other hand, to reduce dust particle adhesion on the optically transparent surfaces, the surface should have a hydrophobic wetting state. Although several methods were introduced to create a hydrophobic wetting state at the surfaces,^20–23^ the method utilizing the deposition of functionalized silica particles is simple, and it offers improved hydrophobic characteristics at the surface, *i.e.*, high contact angle of droplet with low hysteresis. In addition, the optical transmittance reduction remains small after the nanosize particles' deposition on surfaces.^23^ Consequently, in the present study, removal of the environmental dust particles from the inclined optically transparent and hydrophobic surface is examined. Glass surfaces are coated using the functionalized silica particles to create the hydrophobic wetting state on the surface. Environmental dust particles are collected from the local region of Dammam in the Kingdom of Saudi Arabia (KSA), and they are distributed onto the hydrophobic glass surface while mimicking the conditions observed in the local area. An innovative self-cleaning method is introduced that generates the avalanche effect on the hydrophobic surface; in this case, a small amount of zirconium oxide and Inconel 625 powders are locally deposited on the inclined dusty surfaces. The selection of zirconium oxide and Inconel 625 powders is based on their densities, which are higher than the density of dust particles, and sizes, which are larger than the average dust particle size. The dust particle-deposited surface is inclined with a gradually increasing inclination angle, while a high-speed camera is used to observe the dust particles' motion on the surface during the inclinations. The formulation of the particle acceleration on the inclined surface is presented, and findings are compared with those obtained from the high-speed camera data. The dust particle adhesion on the hydrophobic surface is measured, incorporating atomic force microscopy. UV-visible transmittance of the hydrophobic glasses prior to and after inclination tests is also measured.

RETRACTED

## Experimental

Glass samples composed of 76.5% SiO_2_, 9.9% CaO, 1.2 MgO and 12.4% Na_2_O with the dimensions of 30 mm × 100 mm × 1 mm (width × length × thickness) were used in the experiments. The glass surfaces were cleaned in a piranha solution prior to coating with the functionalized nano-sized silica particles. The nano-sized silica particles were obtained *via* a synthesis involving tetraethyl orthosilicate (TEOS), 3-aminopropyltrimethoxysilane (AMPTS), isobutyl(trimethoxy)silane (OTES), ethanol, and ammonium hydroxide. The synthesis process was described in the early study, and the details of the process were referred to.^24^ The solution containing the synthesized silica particles was mixed with the modifier silane molecules having the molar ratio of 3 : 4 in order to functionalize the silica particles. The final solution was stirred for 15 hours at room temperature, centrifuged, and washed with ethanol to remove the reactants in the mixture. The solvent casting technique was adopted to coat the glass surface with functionalized silica particles. In this case, the deep coating was done using a coating unit (Chemat Scientific KW 4AH by Chemat Technology Inc.). The deep coating chamber was set to spin at a constant speed for five minutes, and later, the samples were pulled from the chamber at a constant speed (0.1 mm s^−1^). The coated surface was vacuum dried, ensuring all the solvents were evaporated on the coated surface, which was later characterized. The functionalized silica particles deposited on the glass surface resulted in a uniform hydrophobic wetting state on the surface, with the droplet contact angle of 158° ± 2° and hysteresis of 2° ± 1°.

Soft brushes were used to collect the environmental dust particles from photovoltaic panel surfaces in the local area of Dammam in the Kingdom of Saudi Arabia, and the dust particles collected were stored in a sealed container prior to the experiments. The average of dust particle sizes was measured using the particle size analyzer, and the particles were later characterized using scanning electron microscopy (SEM by JEOL 6460), energy dispersion spectrometry (EDS by JEOL 6460), and X-ray diffraction (XRD by Bruker D8 Advanced with Cu-K_α_ radiation source). Surface texture assessment, including the averaged surface roughness and surface profile, was carried out with the atomic force microscope (5100 AFM/SPM by Agilent). The size of the silicon nitride probe tip was *r* = 20–60 nm, with a manufacturer specified force constant (*k*) of 0.12 N m^−1^. The dust adhesion, in terms of the tangential and frictional forces, on the hydrophobic glass surface was measured, using the atomic force microscope in the friction mode.

RETRACTED

The adhesion of the nano-sized coating on the glass surface was assessed using a linear microscratch tester (MCTX-S/N: 01-04300). In this case, the contact and end loads were kept at 0.03 N and 2.5 N, respectively, and the scanning speed was adjusted at 5 mm min^−1^ with the loading rate of 0.01 N s^−1^. The UV-visible transmittance of the glass surfaces prior to and after experiments was measured with a UV spectrometer (Jenway 67 Series spectrophotometer).

In the experiments, a servomotor-derived precision fixture was designed and realized to tilt the coated glasses with an incremental angle of 0.1°. The dust particles collected were deposited uniformly using the fine-sized metallic meshes (25 μm spacing) on the coated glass surface. The layer thickness of the dust particles was set according to the environmental conditions. In the local environment, the accumulated dust thickness was measured over the period of four weeks, and the dust layer thickness was measured to be in the order of 200 μm. Consequently, in the experiments, the layer thickness of the dust particles was fixed at 200 μm. The actual ambient conditions were simulated in the lab environment, in which case, the test chamber was maintained at constant atmospheric pressure of 101.32 kPa, temperature of 311 K, and relative humidity of 85%.

## Results and discussion

Environmental dust removal from the inclined hydrophobic glass surfaces is investigated, and the influence of the heavy and large particles on the dust removal rate is presented. Functionalized silica particles are deposited on the glass surface to obtain the hydrophobic wetting state; the environmental dust particles are collected from the local region of Dammam in Saudi Arabia.

### Characterization of hydrophobic glass surface and dust particles

Fig. 1a shows the SEM micrograph of the surface coated with nano-sized silica particles. The surface possesses agglomerated silica particles with the presence of few porous-like structures. It is free from large-sized asperities, including voids and cracks. The occurrence of agglomeration of the silica particles is mainly associated with the modifier silane, which causes side reactions and condensation on the silica surface while contributing to the agglomeration.^25^ The pore-like structures do not cover a large area on the surface, and they are not connected with the intermediate scattered small pores. The total area covered by the pore-like structures is in the order of 4% of the total area of the coated surface. However, the pore-like structures can act like air capturing centers while contributing to the texture of the surface. Fig. 1b shows the AFM 3-dimensional micro image of the silica particle-coated surface, while Fig. 1c shows the AFM line scan on the same surface. The presence of nano-sized spherical particles is evident from the 3-dimensional image of the surface (Fig. 1a and b). The agglomerated nano-sized silica particles form a surface texture with the average surface roughness in the order of 90.5 nm. The average depth of the pore-like structures is in the order of 75 nm, which can be observed from the AFM line scanning curve (Fig. 1c); however, the pore-like structures contribute to the surface roughness parameter. In order to assess the free energy of the coated surface, droplet method is adopted.^26^ In this case, the droplet contact angle is measured for water, glycerol, and diiodomethane, in line with the early study.^26^ The details of the surface energy calculations are given in the Appendix. The surface energy of the functionalized nano-sized silica particle-coated surface is in the order of 38.14 mN m^−1^, which is slightly lower than that reported for CVD plasma enhanced tetraethylorthosilicate (PE-TEOS) coated surface (42.12 mN m^−1^).^27^Fig. 1d shows the optical image of the droplet on the functionalized silica particle-coated surface. The contact angle measurements were carried out, adopting the method introduced in the previous study. The water droplet contact angle is in the order of 158° ± 2°, and the contact angle hysteresis is 2° ± 1°. The coated surface has a superhydrophobic wetting characteristic with extremely small hysteresis. The contact angle and its hysteresis remain uniform on the coated surface, with a very small variation. Consequently, the functionalized nano-sized silica particle-coated surface has uniform wetting characteristics, which is associated with the uniformly distributed hierarchal texture structure and almost constant surface free energy. The adhesion of the coating on the surface was assessed through the measurement of the tangential force required to remove the coating from the surface. Fig. 2a shows the tangential force variation along the surface, while Fig. 2b shows the scratch mark on the surface. The frictional force is also included for comparison in Fig. 2a. The tangential force remains considerably higher than the frictional force measured on the coated surface. Consequently, the adhesion between the coated particles on the glass surface remains significantly high. The tangential force measurements were repeated at different locations on the coated glass surface, and findings revealed that the variation in the adhesion work is in the order of 4%. Consequently, the coating attaches at the glass surface with a strong and uniform bonding. The small-sized scratch mark also indicates no peeling of coating from the surface and strong adhesion between the coating and the surface.

RETRACTED

**Fig. 1:** SEM micrograph, AFM image, and AFM line scan of the silica particle-coated surface: (a) SEM micrograph of coated surface, (b) AFM 3-dimensional image of coated surface, (c) AFM line scan on coated surface, and (d) optical image of water droplet on the coated surface.

**Fig. 2:** Tangential and frictional forces along silica particle-deposited surface, and scratch marks left on surface: (a) tangential and frictional forces and (b) microscopic image of scratched surface. Tangential force represents the force required to remove the coating from the surface.

Fig. 3 shows the SEM micrograph of the dust particles. The dust particles collected from the local area have different shapes (Fig. 3a) and sizes (Fig. 3b). Some of the small dust particles attach at the surface of the large particles (Fig. 3b). The small dust attachment is related to the charges developed during the prolonged duration of exposure to solar radiation of the suspended small-sized dust particles in air, particularly near the region of the Gulf sea.

**Fig. 3:** SEM micrographs of dust particles: (a) various shapes of dust particles and (b) small-sized dust particles attached to the larger dust particle surface.

In this case, the interaction of solar irradiation with the small particles during the prolonged exposure results in bonding of some ionic compounds to the dust particles.^1^ The X-ray diffractogram of the dust particles is shown in Fig. 4, while Table 1 provides the dust particles' elemental composition (wt%).

**Fig. 4:** X-ray diffractogram of dust particles.

**Table 1:** Elemental composition (wt%) of dust particles and dried liquid solution

	Si	Ca	Na	S	Mg	K	Fe	O
Dust particles	12.2	8.1	2.1	1.8	0.9	1.1	1.1	Balance

In the X-ray diffractogram, the iron peaks overlay with Si, and they are associated with the clay-aggregated hematite (Fe_2_O_3_). The sulfur peak is related to the anhydrite or gypsum (CaSO_4_) components in the dust. From Table 1, the dust particles comprise various elements, which include Na, K, Ca, S, Si, O, Mg, Fe, and Cl. However, the geologic structure of the local environment can influence the elemental composition of the dust particles collected. In the case of small particles (<1 μm), the concentrations of some elements such as Na, K, Ca, O, and Cl are slightly higher than those of the large particles. This variation may be related to the prolonged duration of suspension of small particles in air, which undergo a long interaction duration with solar radiation. The dust particles' geometry can be grouped by the shape factor (*R*_Shape_), which can be represented as , where *P* represents the dust particle perimeter and the *A* is the total area of the dust particles, and the aspect ratio (*A*_Aspect_), which is , where *L*_Projection_ is the longest projection length of the dust particle.

RETRACTED

The aspect ratio is associated with the approximate roundness of the particle, and it corresponds to the ratio of the major-to-minor axes of an ellipsoid that is best fit to the particle. The shape represents complexity of the particle, and it is the inverse of the particle circularity; however, the *R*_Shape_ of one corresponds to a perfect circular shape. The detailed experimental measurements demonstrate that no functional relation is observed among the particle size, the aspect ratio and the shape factor. An inverse relation occurs between the size of the dust particle and the aspect ratio; however, a direct relation takes place between the size of the dust particle and the shape factor. The particle aspect ratio becomes small once the shape factor becomes large, which is more pronounced for the large dust particles (>5 μm). The shape factor becomes almost one for the small dust particles (<2 μm), and the median shape factor becomes 3 for the large particles (>5 μm). The multiple corners around some of the dust particles act like anchoring sites while influencing the movement of each dust particle, *i.e.*, the movement of the group of dust particles is observed when external force is applied.

### Mechanics of dust particle removal from treated glass surfaces

The dust particles on the inclined surface can move under the influence of gravitational potential energy while satisfying the force balance. The inertia force, which drives the particle movement on the surface, is the result of the balance among the gravitational, retarding and pinning forces. In this case, the force balance results in:

1 *F*_i_ = *F*_g_ sin *δ* − (*F*_Ad_ sin *δ* − *F*_L_ + *F*_f_ + *F*_D_)

where *F*_i_ is the inertia, *F*_g_ is the gravitational force, *δ* is the inclination angle of the surface, *F*_Ad_ is the adhesion force due to interfacial tension between the dust particle and the surface, *F*_L_ is the lift force acting on the dust particle due to the shear flow generated during particle motion, *F*_f_ is the kinematic frictional force, and *F*_D_ is the drag force. On the other hand, the dust particle is pinned to the inclined surface because of the adhesion and frictional forces generated in the plane and normal to the surface. Few models have been introduced to formulate the adhesion of particles on surfaces. In general, the van der Waals force can be considered to be the dominant force in particle adhesion on surfaces in dry and electrodynamically neutral environments.^28^ The model developed by Johnson *et al.*^29^ formulates the adhesion force, incorporating the van der Waals force acting on the spherical particles; however, the model assumes the smooth surfaces of particles and can also be applicable for smooth flat surfaces. The adhesion force (*F*_Ad_) takes the form ; here, *R*_p_ is radius of the particle and *γ*_i_ is interfacial surface energy between two surfaces. The force equation describing the adhesion is limited, with the large soft bodies having a high surface energy.^28^ This model was modified by Derjaguin *et al.*^30^ for small and hard particles with smooth surfaces and low surface energies; in this case, the force equation for adhesion becomes *F*_Ad_ = 2π*R*_p_*γ*_i_, and here the constant is modified. Hamaker^31^ introduced a new model for the formulation of the adhesion force incorporating the particle spacing (distance between the particle and the surface). The equation takes the form , here *A* is Hamaker constant and *Z*_o_ is particle spacing, which is of the same order of separation distance between the particle surface and the flat surface. The adhesion equation can provide a correct estimation of the adhesion force for the particle spacing in the range of 0.3 or 0.4 nm.^28^ Hamaker's model was modified by Rabinovich *et al.*,^32^ introducing the rough surface parameter, which is same order of the root mean square of rough surface texture. The adhesion force yields the form , where *r*_s_ is the surface roughness parameter. Since the coated surface has texture because of the functionalized silica particle deposition (Fig. 1c) and, similarly, the surface of the dust particles are also rough, the model modified by Rabinovich *et al.*^32^ is used to assess the adhesion force between the dust particles and the inclined hydrophobic surface. The dust particles, when moving on the inclined surface, suffer from drag forces, which comprise the frictional and pressure drag forces. The drag force generated on the dust particles is associated with the combination of pressure and shear forces. The drag force for slow-moving particles in shear flow is formulated by O'Neill *et al.*^33^ and Goldman *et al.*,^34^ while incorporating the spherical particle in the momentum equation (Navier–Stoke equation). The formulation yields the drag force in the form of *F*_D_ = *C*_d_π*μ*_f_*R*_p_*u*_f_, where *C*_d_ is the drag coefficient, *μ*_f_ is the fluid viscosity, which is air, and *u*_f_ is the flow velocity around the particle. The drag coefficient is considered as 0.3 in the analysis. Since the shear flow is created by the motion of the dust particles on the inclined hydrophobic surface, it is assumed that the shear flow velocity is of same order as the particle velocity. The motion of the dust particles on the inclined surface can also create a lifting force in the shear flow. The analysis for the spherical particle lifting in shear flow has been done earlier.^35^ The lift force normal to the inclined hydrophobic surface is: ,^35^ where *C*_L_ is the lift coefficient,  is the fluid strain, and *L* is the normal distance between the inclined surface and the particle center. After assuming that the particle and surrounding air have the same velocity and flow behaviour, similar to coquette flow in the shear layer, the drag coefficient can be obtained from the data presented in the previous study.^35^ The local Reynolds number (, where *υ*_f_ is the fluid kinematic viscosity) of the particle in shear flow, remains critical to obtaining the lift coefficient from the data.^35^ The direction of the lift force is opposite to the direction of the adhesion force, and the lift force lowers the dust particle adhesion on the surface during its motion. Moreover, the kinetic friction force is associated with the friction coefficient between the dust particles and the inclined surface during the dust particle motion. This can be written as *F*_f_ = *μ*_d_*mg*, where *μ*_d_ is the kinetic friction coefficient, which can be determined from the atomic force microscopy measurements.

RETRACTED

Therefore, the dust particle acceleration on the inclined surface can be obtained from eqn (1), which yields:2where *m*_p_ is the mass of the dust particle. In order for the dust particle to overcome the retarding and pinning forces, the condition of  should be satisfied. The velocity of the dust particle on the inclined surface can be obtained from integration of the acceleration along the time, *i.e.*, integration of eqn (2) yields:3

In order to assess the adhesion force and the kinetic friction coefficient, force measurements using the atomic force microscope were carried out. Fig. 5a shows the atomic force microscope image of the dust particle on the coated surface, while Fig. 5b shows the tangential force obtained from the atomic force microscope tip (in mV unit), under the friction mode, when the dust particle is moved on the surface. The force corresponding to the initial peak is associated with the adhesion and the friction forces, and the remaining peaks along the displacement are related to the frictional forces between the dust particle and the coated surface. However, the atomic force microscope cantilever tip sensitivity is related to the slope of the deflection of the tip while the tip is in contact with the surface. From the deflection relation, the adhesion force can be written as: *F* = *kσ*Δ*V*, where *k* is the spring constant of the cantilever tip (N m^−1^), *σ* is the slope of the displacement over the probe voltage recorded (Δ*z*/Δ*V*, m V^−1^), and Δ*V* is the voltage recorded during the surface scanning by the tip in contact mode. In the measurements, the following data is adopted from the calibration of the atomic force microscopy tip: *kσ* = 2.45456 × 10^−16^ N mV^−1^. In this case, the adhesion force obtained from the atomic force microscopy measurement is in the order of 1.1 × 10^−5^ nN. It should be noted that the average density of the dust is in the order of 2800 kg m^−3^, and the dust size used to measure the adhesion force is in the order of 1.15 μm (Fig. 5a). Moreover, the adhesion force calculated from the Rabinovich relation . For 1.15 μm dust particle size, which is close to the average dust particle size (1.2 μm), is in the order of 4.3 × 10^−5^ nN. The difference between the adhesion force obtained from the measurements and the prediction using the Rabinovich relation is associated with the assumptions made in the model, which consider the circular shape of the particle; however, the dust particle does not possess an exactly circular shape. In addition, the experimental errors contribute to this difference, which is estimated to be in the order of 10%. It should be noted that AFM measurements are repeated seven times, incorporating the various sizes of the dust particles. The findings reveal that the error estimated based on the experimental repeatability is in the order of 10%. The kinetic friction coefficient between the dust particle and the hydrophobic surface, as determined from the atomic force microscopy data, is in the range of 0.15–0.120 ± 0.006. The force balance equation (eqn (2)) reveals that the particle acceleration on the surface is in the order of 7.783 m s^−2^.

**Fig. 5:** 3-Dimensional AFM image and friction data for dust particles on the surface and frictional force along the scanning line obtained during dust particle movement: (a) 3-dimensional AFM image of dust particles, (b) 3-dimensional frictional force data, and (c) force data along the surface during dust movement by AFM tip. Force unit is in mV.

RETRACTED

The force generated by the gravitational acceleration due to a single dust particle is 7.072 × 10^−4^ nN; the adhesion, friction, and drag forces are in the order of 1.1 × 10^−5^ nN, 1.11 × 10^−4^ nN, and 3.3 × 10^−4^ nN, respectively. The dominant force during the particle motion on the inclined surface is the gravitational acceleration, and the dust particle retarding/pinning forces in terms of adhesion, friction, and drag are almost of the same order. The lifting force is found to be almost 7% of the adhesion force, which does not significantly influence the force balance equation (eqn (2)). Fig. 6 shows the optical image of the dust particles on the inclined surface at various times, while Fig. 7 shows the velocity of the dust particles obtained from the experiment along the hydrophobic surface when the inclination angle of the hydrophobic surface is 60°, at which the dust particles initiate moving on the inclined surface. The velocity remains low during the early movement of the dust particles on the inclined surface. As the distance along the inclined surface increases, the dust particles accelerate and the velocity increases sharply. However, the velocity increase becomes gradual as the distance further increases on the inclined surface. In this case, the dust particles almost attain a steady movement on the surface. The dust particle velocity obtained from eqn (3) is in the range of 0.11–0.25 m s^−1^, which is slightly higher than that obtained from the experiment. This difference is because of the experimental errors, which are estimated to be in the order of 10%, the assumption of spherical dust particles in the analysis, and the error involved with the estimation of the friction coefficient and the adhesion force calculations, which is in the order of 10%. Nevertheless, the analytical formulation provides a similar velocity trend with that obtained from the experiments. In order to accelerate the particle removal and increase the area of the dust removed from the surface, avalanche influence is introduced. In this case, high density particles, such as zirconium oxide (*ρ* = 5680 kg m^−3^) and Inconel 625 (*ρ* = 8440 kg m^−3^) powders, which are heavier than the dust particles (*ρ* = 2800 kg m^−3^), are located on the top region of the hydrophobic glasses covered by the dust particles.

**Fig. 6:** Optical images of dust particle displacements at various times on the inclined hydrophobic surface. Inclination angle is 60°.

**Fig. 7:** Velocity of dust particles along the inclined hydrophobic surface. Inclination angle is 60°.

The hydrophobic glass is later tilted to observe the motion of the heavy and dust particles on the surface *via* using a high speed camera. In order to assess the effect of the coverage area of the heavy particles on the dust removal rate from the surface, three different sizes of coverage area of the heavy particles are introduced on the hydrophobic glass surface (Fig. 8a). The coverage area of the heavy particles varies between 35.05 m^2^ and 14.65 m^2^. Fig. 8b shows the surface of the glass after tilting the surface at the angle of 40.5°. The dust particles on the glass surface remain after tilting, except the dust particles in regions where the high density particles are situated. Consequently, the gravitational potential energy enables movement of dust particles on the hydrophobic surface under the influence of high density particles. It should be noted that high density particles are subjected to higher gravitational force than the dust particles because of their high density, which initiates early movement of the particles on the surface at lower inclination angle than that corresponding to the case of only dust particles on the surface. The movement of the high density particles creates the avalanche effect on the inclined surface, and the surface area where the dust particles are removed remains larger than the projection area of the high density particles on the surface.

RETRACTED

**Fig. 8:** Optical images of the dusty hydrophobic surface with the presence of high density particles prior to and after tilting: (a) high density particles and dusty surface prior to tilting, and (b) high density particles and dusty surface after inclining at 60°.

The area ratio of the dust removed surface over the area of the high density particles on the surface is given in Table 2 for zirconium oxide and Inconel 625 powders. The inclination angle of the hydrophobic surface is 40.5°. Increasing high density particle size enhances the area where the dust particles are removed from the surface. However, reducing the area of the high density particles on the hydrophobic surface enhances the area ratio of dust removed surface over the area of high density particles, which is true for zirconium oxide and Inconel 625 particles. This indicates that the area removed from the dust particles is not a linear function of the area coverage of the high density particles. Fig. 9 shows the velocity of the high density particles along the inclined surface for three different coverage areas of the high density particles. The inclination angle of the hydrophobic surface is 40.5°. The rise of the velocity of Inconel 625 particle is rapid, and increasing the area of the particles initiates the early movement of the particles from the inclined hydrophobic surface (Fig. 9a). As the coverage area of the particles reduces, some small delay occurs for the initiation of the Inconel 625 particle movement from the surface. In this case, increasing the coverage area of the Inconel alloy powders results in early movement of the particles from the inclined hydrophobic surface under the influence of the gravitational potential energy. The maximum velocity of Inconel particles reaches almost 0.14 m s^−1^ in the bottom region of the inclined hydrophobic glass surface. In the case of zirconium powders (Fig. 9b), the rise of velocity is sharp in the early period, becoming gradual with progressing time. This behaviour is true for all the coverage areas of zirconium oxide particles tested on the inclined surface. Similarly, reducing the coverage area of zirconium particles gives rise to delay in the initiation of falling of the particles from the inclined hydrophobic surface. The maximum velocity of zirconium oxide particles is in the order of 0.12 m s^−1^, which is slightly lower than that corresponding to Inconel 625 powder. The previous formulation for the avalanche velocity can be used to predict the velocity of the dust particles when the high density particles are used. Hence, in line with the early study,^36^ the avalanche velocity along the inclined surface can be written as: , where *η* is the eddy viscosity, *h* is the dust film thickness on the inclined hydrophobic surface, *g* is the gravitational acceleration, *s* is the distance along the inclined surface, and *δ* is the inclination angle. Incorporating the data, *η* = 1000 m s^−2^,^36^*h* = 100 μm, and *δ* = 40.5°, the avalanche velocity for *s* = 3 cm distance on the inclined surface becomes in the order of 0.11 m s^−1^, which is close to the value measured from the experiments (0.14 m s^−1^ for Inconel 625 or 0.12 m s^−1^ for zirconium oxide).

RETRACTED

**Table 2:** Area of the zirconia and Inconel particles on the glass surface prior to inclination of the glass

Zirconium oxide powder			Inconel 625 powder		
Powder area (mm^2^)	Dust removed area	Area ratio	Powder area (mm^2^)	Dust removed area	Area ratio
28.30	135.57	3.488	35.05	101.60	2.90
24.30	128.82	5.31	28.09	85.60	3.05
14.65	122.03	8.33	16.33	75.40	4.62

**Fig. 9:** Velocity of high density particles along the inclined surface at 60° inclination angle with the presence of ZrO_2_ and Inconel 625 powders: (a) ZrO_2_ particles, (b) Inconel 625 particles. Avalanche effect is created with high density particles on the inclined hydrophobic surface to enhance dust particle removal from the surface.

The dust particle-removed hydrophobic surfaces were tested optically by measuring the UV-visible transmittance of the surfaces. Fig. 10 shows the UV-visible transmittance of the normal glass, silica particle-coated glass, dusty glass, and dust particle-removed glass. The silica nano-sized particle coating reduces the optical transmittance of the surface; however, the optical transmittance reduces significantly after covering the coated surface with the dust particles. The optical transmittance increases notably after the dust particles are removed from the hydrophobic surface. Although the optical transmittance of the dust-removed surface remains slightly lower than that of the coated surface, it improves significantly as compared to the dusty hydrophobic surface. The reduction in the optical transmittance of the dust-removed surface is associated with the small dust residues remaining on the surface, which can be observed from Fig. 11, in which SEM micrographs of the dust residues on the hydrophobic surface is shown. The dust particle residues are small in size and appear in odd shapes (Fig. 11a and b). Energy dispersive spectroscopy (EDS) analysis of the dust residues reveals that the oxygen content in these residues is large, almost twice that of the original dust particles. This demonstrates that the dust residues have low mass density, which is estimated as 1200 kg m^−3^ from the EDS data. Consequently, the gravitational potential energy initiating the removal of these particles on the inclined surface is not sufficiently high to overcome the pinning forces, despite the high density particles used to create the avalanche influence. In addition, some of the edges of these particles are sharp (Fig. 11), and it is possible that these particles anchor the surface texture and possibly mechanically attach to the surface.

**Fig. 10:** UV visible transmittance of as received glass surface, silica particle coated; dusty; and dust particle-removed, silica particle-coated surface *via* inclining at 60°.

**Fig. 11:** SEM micrographs of dust residues on coated surface after dust removal from 60° inclined hydrophobic surface: (a) small size particles with high oxygen content (light particles), and (b) sharp edges particles.

## Conclusion

Removal of dust particles from the hydrophobic optically transparent glass surfaces is considered. The hydrophobic wetting state of the glass surfaces is achieved through coating the glass surface with functionalized nano-sized silica particles. The avalanche effect is created to enhance the dust particle removal rate from the surface. The hydrophobic surface is inclined, and the particles with higher density than the density of the dust particles are introduced locally on the dust-deposited inclined surfaces. The dynamics of the dust particles on the inclined surface, together with the influence of the high density particles on the dynamics of dust particle removal from the surface, are examined. An experiment is carried out with the high speed camera to measure the velocity of the dust particles on the inclined hydrophobic surface. The predictions of the acceleration of the dust particles and velocities are validated through the experimental data. The optical transmittance of the dust-removed surfaces is measured, and the geometric features and elemental composition of the dust residues on the dust-removed surfaces are assessed. The findings revealed that the predictions of the acceleration and velocities of the dust particles agree well with the experimental findings. The hydrophobic wetting state of the surface improves dust removal from the surface *via* surface inclination. The inclusion of high density particles (zirconium oxide and Inconel 625 powders), which have higher density than the dust particles (2800 kg m^−3^), creates an avalanche effect on the inclined surface while initiating the dust removal at a small inclination angle of the surface. The inclination of the hydrophobic surface for the initiation of dust particle removal is in the order of 60°; however, this angle reduces to 40.5° as the high density particles are localized on the dusty hydrophobic surface. The area from which the dust particles are removed increases with the amount of high density particles on the surface; however, no simple functional relation is observed between the coverage area of the high density particles and this area. On the other hand, the dust particles are composed of various elements, including alkaline and alkaline earth metals, sulphur, iron, chlorine, and oxygen. Some small dust particles attach at the surface of the large size dust particles while forming clusters. Some dust residues are observed on the inclined surface after the dust particles are removed under the avalanche influence. The dust residues have, mainly, sharp edges and high oxygen content. The sharp edges of the dust particles partially anchor the surface texture generated by the functionalized silica particles, and the presence of high oxygen content lowers the density of the dust particle residues. In this case, the avalanche influence generated could not remove these dust particles from the inclined hydrophobic surface. The UV visible transmittance of the dust particle-removed surface improves considerably as compared to that of the dusty surface.

RETRACTED

## Appendix: droplet method for formulation of surface free energy

The assessment of the surface free energy of solids and liquids was introduced earlier by van Oss *et al.*^26^ This can be written as:

4 *γ* = *γ*^L^*+ γ*^P^

where *γ*^L^ is the apolar component due to Lifshitz–van der Waals intermolecular interactions and *γ*^P^ is attributed to electron-acceptor and electron donor intermolecular interactions. The apolar component *γ*^P^ owing to electron-acceptor and electron donor intermolecular interactions can be expressed as:^26,37^5where *γ*^+^ and *γ*^−^ are the electron acceptor and electron donor parameters of the acid–base component of the solid and liquid surface free energy, respectively. The interfacial free energy for a solid–liquid system can be expressed as:^26,37^6where subscripts S and L represent solid and liquid phases, respectively. Young's equation for the surface free energy of a solid becomes:^37^

7 *γ*_L_ cos *θ* = *γ*_S_ − *γ*_SL_ − Pe_L_

where *γ*_S_ is the solid surface free energy, *γ*_SL_ is the interfacial solid–liquid free energy, *γ*_L_ is the liquid surface tension, *θ* is the droplet contact angle, and Pe_L_ is the pressure of the liquid film, which is negligibly small and considered to be zero.^26^ Combining eqn (6) and (7) and re-arranging them yields:8

Eqn (8) can be incorporated towards the evaluation of *γ*^L^_S_, *γ*_S_^+^, and *γ*_S_^−^ while using the contact angle data and *γ*^L^_S_, *γ*_S_^+^, and *γ*_S_^−^. The data for *γ*^L^_S_, *γ*_S_^+^, and *γ*_S_^−^ can be found from the literature for water, glycerol, and diiodomethane, which are given in Table 3.^38^ The contact angle measurements were repeated five times to ensure the measurement repeatability of the data in line with the previous study.^39^

**Table 3:** Lifshitz–van der Waals components and electron-donor parameters used in the simulation^26,38^

	*γ*_L_ (mJ m^−2^)	*γ* ^L^_S_ (mJ m^−2^)	*γ*_S_^+^ (mJ m^−2^)	*γ*_S_^−^ (mJ m^−2^)
Water	72.8	21.8	25.5	25.5
Glycerol	64	34	3.92	57.4
Diiodomethane	50.8	50.8	0.72	0

## Conflicts of interest

There are no conflicts to declare.

## Supplementary Material
